# Effects of Long-Term Vagus Nerve Electrical Stimulation Therapy on Acute Cerebral Infarction and Neurological Function Recovery in Post MCAO Mice

**DOI:** 10.1155/2022/8131391

**Published:** 2022-03-29

**Authors:** Li Du, Zhenxing Yang, Huaxin Sheng, Min Liu, Qian Sun

**Affiliations:** ^1^Department of Anesthesiology, Renmin Hospital of Wuhan University, Wuhan, China; ^2^Department of Neurosurgery, Renmin Hospital of Wuhan University, Wuhan Hubei, China; ^3^Multidisciplinary Neuroprotection Laboratory, Department of Anesthesiology, Duke University Medical Center, Durham, USA

## Abstract

**Background:**

Vagus nerve stimulation therapy is proven to produce neuroprotective effects against central nervous system diseases and reduce neurological injury, having a positive effect on the recovery of neurological functions in mouse model of stroke.

**Objective:**

This study was aimed at exploring a wider time window for VNS treatment, investigating the long-term behavioral improvement of long-term VNS in mice after pMCAO, and exploring the antiapoptotic properties of VNS and its role in autophagy, all of which may be a permanent deficiency potential mechanism of neuroprotection in hemorrhagic stroke.

**Methods:**

Permanent focal cerebral ischemia and implantation of vagus nerve stimulator were performed through intracavitary occlusion of the right middle cerebral artery (MCA). The vagus nerve stimulation group received five times vagus nerve stimulation from 6 h after surgery for 5 days. Adhesive removal test and NSS neurological score were used to evaluate the neurological deficit of mice. TTC staining of mouse brain tissue was performed one week after surgery in order to assess the area of cerebral infarction. Additionally, frozen sections were stained with Fluoro-Jade B to observe the apoptotic cells in the ischemic penumbra of brain tissue. Finally, Western blot was used to detect the changes in the levels of apoptosis-related proteins such as cleaved-caspase3 and Bcl-2 and autophagy-related proteins such as mTOR, Beclin-1, and LC3-II in brain tissue.

**Results:**

VNS can effectively reduce the behavioral score of pMCAO mice; TTC results showed that VNS could effectively reduce the infarct area after pMCAO (*P* < 0.05). After VNS intervention of the pMCAO group compared with the pMCAO+VNI group, the FJB-positive cells in the VNS group were significantly decreased (*P* < 0.05); Western Blot analysis showed that the expression of cleaved-caspase3 in the brain tissue of mice increased after pMCAO (*P* < 0.05), and the expression of Bcl-2 decreased (*P* < 0.05). This change could be effectively reversed after VNS intervention (*P* < 0.05).

**Conclusion:**

VNS could effectively improve the behavioral performance of mice after permanent stroke in addition to significantly reducing the infarct size of the brain tissue. The mechanism may be related to the effective reduction of cell apoptosis and excessive autophagy after pMCAO by VNS.

## 1. Introduction

Stroke is the second leading cause of death globally and is one of the main causes of disability. Due to the aging among the general population, the incidence is increasing on an annual basis [1]. Meanwhile, as the proportion of unhealthy eating habits increases, the proportion of young people suffering from stroke is also increasing [2]. Intravascular interventional thrombolysis and anticoagulants are still the backbone of treatment worldwide. However, due to the limitation of the interventional treatment time window, the proportion of patients treated within a suitable time frame is limited to 10% or less. Drug thrombolytic therapy has serious complications such as hemorrhage, and the treatment effect for stroke is not ideal. Nerve stimulation is an alternative or auxiliary method for the treatment of failed thrombolysis, which in turn can protect the brain during acute ischemia. In addition, nerve stimulation can also repair the nerve function of patients (treated or untreated) with severe functional impairment in the poststroke stage in addition to promoting the recovery of neuronal function. In the past few decades, various animal stroke models have shown the efficacy and safety of many candidate neuroprotective agents, but in clinical trials, promising preclinical studies have not yet been translated into positive results [3].

Ideally, the future treatment plan for ischemic stroke should include thrombolysis, antithrombosis (secondary prevention), neuroprotection (stabilizing penumbra), and strategies to enhance neuroplasticity.

Vagus nerve stimulation is proven to play a potential protective role in central nervous system diseases such as Alzheimer's disease and traumatic brain injury [4, 5]. It has been suggested to provide protection against ischemic brain injury. So far, however, the vagus nerve stimulation experiment reported in the relevant paper was a single stimulation during or after surgery, and there are no further researches on the long-term stimulation of the vagus nerve on the recovery of nerve function after cerebral ischemia. We have designed a new vagus nerve stimulation therapy with a wider time window that can observe the effect and the change of the electrical stimulation of vagus nerve after brain stroke, which is more in line with clinical needs of achieving neuroprotection.

Ischemic neurons showed both necrotic and apoptotic features [6]. The same neurons also exhibited caspase-3 cleavage and cytochrome-C release as markers of apoptosis. It seems that Bcl-2 family protein members play a key role in mediating necroptosis by inducing necrotic mitochondrial damage [7]. The signaling pathway of autophagy is driven on mechanistic target of rapamycin (mTOR), which leads to autophagy initiation, respectively [8]. We plan to evaluate the protective effect of vagus nerve stimulation on cerebral ischemia injury in mice by analyzing the changes in the above proteins and signaling pathways.

## 2. Materials and Methods

### 2.1. Ethics Statement and Animals

Animal experiments were carried out in accordance with the Duke University Animal Care and Use Committee. All studies were approved by the United States Public Health Service's Policy on Humane Care and Use of Laboratory Animals. Inbred male C57BL6/J mice, 12-14 weeks old (Jackson Laboratories, Bar Harbor, ME). The online tool QuickCalcs (http://www.graphpad.com/quickcalcs/) was used to randomly assign animals to groups.

### 2.2. pMCAO Model Establishment

The pMCAO mice model are made as the article described as follows [9]. The mice were anesthetized with isoflurane, intubated, and ventilated. Their rectal temperature was maintained at 37°C ± 0.2°C throughout the procedure. Mice were placed in left lateral position, and a small skin incision was made between the right eye and ear. The temporal muscle was cut slightly using a high temperature loop, and a 3 mm long segment of the zygomatic arch was removed. After exposing the skull base and trigeminal nerve branch, a small bone window (3-4 mm^2^) was drilled on the skull above the MCA. The MCA trunk was lifted with an 8-0 needle and permanently ligated with silk suture proximal to the cortical branch to the frontal cortex. The muscle and skin were then closed separately. Animals that did not show an infarct lesion were excluded. 80 male C57BL/6J mice were randomly divided into four groups: (1) sham+VNS group (sham operation+vagus nerve stimulation group), (2) pMCAO+VNS group (pMCAO+vagus nerve stimulation group), (3) pMCAO+VNI group (pMCAO+vagus nerve isolation group), and (4) sham group (sham operation group).

### 2.3. Vagus Nerve Electrode Implantation

An incision was made in the middle of the neck of the mouse to separate the sternohyoid and sternomastoid muscles longitudinally and is then pulled to the side to expose the common carotid artery and the right vagus nerve located outside the carotid sheath. In order to reduce the collateral circulation compensation and ensure the success rate of the middle cerebral artery ischemia model, we ligated the common carotid artery with silk thread. The vagus nerve is carefully separated from the surrounding connective tissue and sympathetic nerve trunk. After the 5 mm long VN is exposed, the exposed end of the VN stimulation electrode is wrapped around the nerve in a spiral form and separated from the surrounding tissue by a rubber sheet. Through a continuity test using an ohmmeter, the contact between the electrode and the exposed VN was intact. The electrode lead is then passed from the tunnel through the fascia to the back of the skin on the neck. In order to prevent the nerve or electrode from shifting, a suture outside of the electrode was done on the skin of the neck (image A-C).

Mice in the pMCAO+VNS group were stimulated with 500 *μ*s width 1 mA electric pulses for 10 min at 5 Hz every day for 10 mins, from 6 h after surgery and each day for 5 days, 5 times in total [10]. The criterion for a successful vagus nerve stimulation is an increase in heart rate variability. Animals that did not show an increased heart rate variability were excluded. Mice returned to standard diet after five days of liquid diet.

### 2.4. Behavioral Test

All evaluations were performed by observers who were blinded to group assignment.

### 2.5. Adhesive Removal Test

All mice were pretrained on the adhesive removal tasks 3 days prior to the VN surgery. The adhesive removal test measures sensorimotor function as previously described [11]. Two small adhesive dots were placed on forepaws, and the amount of time (seconds) needed to contact and remove the sticker from each forepaw was recorded. Recording was then stopped if the animal failed to contact the sticker within 2 min. The test was performed 3 times per mouse, and the average time was used in the analysis before stroke in addition to 7, 14, and 21 days after stroke.

### 2.6. mNSS Test

Mice were tested and scored for neurological deficits using a modified Neurological Severity Score (mNSS) 7, 14, and 21 days after the onset of ischemia. An 18-point neurological score was employed with slight modifications described before [12]. The score consists of 5 individual clinical parameters, including tasks on motor function, alertness, and physiological behavior, whereby 1 point is given for failure. A maximum NSS of 18 point indicates severe neurological dysfunction with failure at all tasks.

### 2.7. TTC Staining

Infarct volume was measured using the 2,3,5-triphenyltetrazolium chloride (TTC) staining method. Brain tissue was removed and frozen at −20°C for 30 min and then cut into 1 mm thick coronal sections (7 slices) and incubated in 2% TTC (Sigma-Aldrich, Saint Louis, MO, USA) at 37°C for 30 min. Each section was soaked in 4% paraformaldehyde for 24 h and was then scanned. ImageJ software was used to analyze the infarct area [13]. All evaluations were performed by observers who were blinded to group assignment.

### 2.8. Fluoro-Jade B Staining

The procedure of Fluoro-Jade B stain is as described in the previous article [14]. Brain sections were mounted on microscope slides and placed in 70% ethanol and ultrapure water for 3 min followed by 3 washes in ultrapure water for 1 min each rinse. Sections were oxidized by soaking in a solution of 0.06% KMnO_4_ for 15 min and then washed 3 times in ultrapure water 1 min each. Sections were subsequently stained in 0.001% Fluoro-Jade B (Sigma-Aldrich, Saint Louis, MO, USA) in 0.1% acetic acid for 20 min. Slides were subsequently washed 3 times in ultrapure water for 1 min each and dried overnight at room temperature. Dried slides were cleared in xylene and coverslips were mounted using paramount.

In this study, four fields of view were randomly selected and photographed in the cerebral cortex infarcted ischemic area in each slice by a fluorescence microscope (Zeiss, Germany). Then, the number of positively stained cells in each field of view was calculated at a higher magnification (200x) by researchers that were blinded to experiment design.

### 2.9. Western Blotting

Western blot analysis was performed as previously described [15]. The concentration of proteins was determined by using a protein assay kit (Bio-Rad, USA). 40 *μ*g of proteins was electrophoresed on SDS-PAGE gels and then transferred onto polyacrylamide difluoride (PVDF) membrane (Millipore, Massachusetts, USA). Membranes were incubated with respective primary antibodies (cleaved-caspase-3, 1 : 1000, Abcam; Bcl-2, 1 : 1000, Thermo Fisher; mTOR, 1 : 2000, Abcam; beclin-1, 1 : 1000, Thermo Fisher; LC3II, 1 : 1000, Thermo Fisher) overnight at 4°C, followed by incubation with horseradish peroxidase- (HRP-) conjugated goat anti-rabbit (1 : 5000, Thermo Fisher) or goat anti-mouse IgG secondary antibodies (1 : 10000, Thermo Fisher) for 1 hour at room temperature. Protein bands were visualized by an enhanced chemiluminescence system (ECL kit, GE Healthcare, USA). Quantification of band intensity was analyzed using ImageJ software. *β*-Actin (1 : 5000, Thermo Fisher) served as loading condition.

### 2.10. Statistical Analysis

All data analyses were performed with Prism 8. Statistical analysis was assessed by unpaired Student's *t*-test (infarct volumes and protein levels) or Mann-Whitney *U* test (neurologic scores and FJC positive cells). Data are presented as mean ± SEM, mean ± SD, or the median. The level of significance was set at *P* < 0.05.

## 3. Results

### 3.1. VNS Treatment Improves Long-Term Behavior Performance in pMCAO Mice

To determine whether VNS treatment promoted neurological recovery in pMCAO mice, mNSS and adhesion removal tests were performed. Compared with the sham operation group and the sham operation+VNS group, ischemic mice (pMCAO+VNS and pMCAO+VNI) performed poorly in behavioral tests at different time points after pMCAO (*P* < 0.05, Figures 1(a)–1(c)). The mNSS score of the sham operation group was zero at each time point (Figure 1(a)), but at 7, 14, and 21 days after pMCAO, the mNSS score of mice in the pMCAO+VNS group was lower than that of the pMCAO+VNI group score (*P* < 0.05, Figure 1(a)). The pMCAO+VNS group had a significantly less time in both contact and remove time (Figures 1(b) and 1(c)) at 7, 14, and 21 days after pMCAO compared to the pMCAO+VNI group (*P* < 0.05). In general, these results suggest that VNS treatment promoted the recovery of neurological function in mice after stroke and significantly improved their limb gratitude and motor function (*P* < 0.05).

### 3.2. VNS Treatment Reduces Cerebral Infarction Volume and Promotes Neuron Survival in pMCAO Mice

As the result of improved neurological function may be attributed to the decrease of the damaged area of brain tissue, the cerebral infarct volume was evaluated by TTC staining (Figures 2(a) and 2(b)). The results showed that VNS treatment significantly reduced the infarct volume compared to the pMCAO+VNI group (*P* < 0.05, Figures 2(a) and 2(b) ). No infarct change was found in the sham group.

### 3.3. VNS Treatment Decreased Neuronal Apoptosis in the Peri-infarct Cortex

Fluoro-Jade B was used as a high affinity fluorescent marker for the localization of neuronal apoptosis to observe in the peri-infarct cortex. In the pMCAO+VNS group, the number of FJB-positive cells significantly increased compared with the pMCAO+VNI group (*P* < 0.05). While the sham group had no significant positive cells (Figures 3(a) and 3(b)). These results suggested that VNS treatment reduces apoptosis in pMCAO injury.

### 3.4. Apoptosis Protein Levels in Brain Tissues of Four Groups of Mice

In order to further investigate whether VNS treatment inhibits neuronal apoptosis in the peri-infarct cortex, we tested the expression levels of cleaved caspase-3 and Bcl-2 in the peri-infarct cortex of the four groups of mice. Statistical analysis was assessed by unpaired *t*-test. Western blot results showed that the Bcl-2 protein level of the VNS-treated group was significantly increased, while the expression of cleaved caspase3 decreased compared with the pMCAO+VNI group (*P* < 0.05, Figures 4(a) and 4(b)).

### 3.5. Autophagy Protein Levels in Brain Tissues of Four Groups of Mice

To further confirm the role of VNS treatment in autophagy-related pathways, we tested the autophagy-related proteins including mTOR, Beclin-1, and LC3II in the peri-infarct cortex. Statistical analysis was assessed by unpaired *t*-test. Western blot results showed that Beclin-1 and LC3II levels were significantly decreased following VNS treatment compared with the pMCAO+VNI group (*P* < 0.05, Figures 5(a)–5(c)), while mTOR expressions were increased compared with the pMCAO+VNI group (*P* < 0.05).

## 4. Discussion

In our research, vagus nerve electrode stimulators were implanted to stimulate the vagus nerve 6 hours after acute cerebral infarction in the mouse model, once a day for five days, which can be used to observe the effects of electrical stimulation of the vagus nerve in mice for a longer period of time. We found that VNS decreased the number of apoptotic cells in the penumbra compared with the pMCAO+VNI group in FJB results. We have also found that VNS treatment increased the Bcl-2 expression and decreased cleaved caspase-3 expression in the peri-infarct cortex. Our results also indicated a decreased Beclin-1 and LC3II, while the expression of mTOR increased compared with the pMCAO+VNI group. The results above indicated that neuroprotection induced by VNS is partly attributable to the inhibition of neuronal apoptosis in the ischemic penumbra and suggested that reduction of neuronal apoptosis and a moderate activation of autophagy in the peri-infarct cortex induced by VNS treatment may be the possible mechanism underlying its neuroprotective effect. The behavioral improvement of pMCAO mice by VNS may be related to its reduction of cell apoptosis with a moderate increase in autophagy.

At present, a relevant paper reports that electrical stimulation of the vagus nerve can in fact reduce the inflammatory response and brain edema in the brain tissue of the mouse after acute stroke and promote the recovery of the neurological function of the mouse with chronic stroke in addition to improving the living ability of the mouse [16, 17]. However, the current electrical stimulation in the paper is a single electrical stimulation that is given immediately after the operation and cannot interfere with the subsequent stroke development process in mice. The inflammatory progression and edema of acute stroke are usually developed gradually a few hours after acute brain stroke. At the same time, long-term animal experiment observation can also provide scientific data and theoretical basis for clinical development of vagus nerve electrical stimulation for the treatment of human acute stroke. In this study, the time window of vagus nerve stimulation therapy was innovatively extended to three days after stroke. From a clinical application perspective, the treatment time window has been effectively extended, and the scope of adaptation is wider, which can allow more strokes to be treated and is expected to restore nerve function to the greatest extent possible.

Previous studies have shown that the appropriate activation of autophagy appears to be beneficial in poststroke conditions, which can remove necrotic materials in tissues. However, the decrease or increase of autophagy protein indicates that the autophagy response is excessive, which will increase the prodeath effect on neuronal cells. Several studies have revealed that autophagy is activated in the penumbra [18, 19]. Here, our results demonstrate that VNS can indeed induce the regulation of autophagy activation in pMCAO mice. Some studies have reported that autophagy is an intracellular protective mechanism, which has been shown to be closely related to inflammation in mice with cerebral ischemia. The activation of autophagy can help the body effectively remove necrotic cells and substances. After ischemia, a large number of neurons and glial cells are ischemic necrosis, and autophagy regulates the inflammatory response. Both respond to the stimulation caused by cerebral ischemia injury [20]. They found that inhibition of autophagy with Beclin-1 siRNA increased the inflammatory response of the main microglia of cells cultured with GSK-3*β* inhibitors in vitro, thereby increasing neuronal damage. Other researchers treated pMCAO mice with the autophagy inhibitor 3-MA and found that the inflammatory response caused by ischemia was alleviated, while the autophagy inducer rapamycin significantly promoted the inflammatory response [21]. In conclusion, our research shows that through the regulation of phagocytic response in mice by VNS, reducing the occurrence of inflammation, reducing neuronal cell apoptosis, and inhibiting glial cell overreaction are potential target therapeutic approaches to reduce brain injury after cerebral ischemia.

Another current explanation for the neuroprotective mechanism induced by VNS is the regulation of the afferent vagus nerve pathway. The afferent nerve activity is relayed to the nucleus tractus solitarius which has projections to the locus coeruleus (LC) [22] and is likely to play an important role in VNS therapy through the release of norepinephrine (NE) and 5-hydroxytryptamine (5-HT) [23]. VNS can activate NE to play the anti-inflammatory effects, which can stimulate the 5-HT releasement [24, 25]. The influence of these afferent nerve pathways may contribute to the effectiveness of VNS in cerebral ischemia. Another suggestive mechanism of neuroprotection induced by VNS is by affecting the efferent vagus nerve pathway. Studies have found that the cholinergic anti-inflammatory pathway (CAP) can be activated by the central cholinergic system of the brain through the stimulation of the efferent fibers of the vagus nerve [26], which is mediated by *α*7 nicotinic acetylcholine receptors. Therefore, CAP plays a key role in the inhibition of inflammation [27], and repeated electrical stimulation of the efferent fibers of the vagus nerve in our experiment may activate the cholinergic anti-inflammatory pathway and reduce the inflammatory response caused by stroke, thereby achieving brain protection The effect of this is consistent with our experimental results, but the specific mechanism needs to be further studied and confirmed.

Although regulatory mechanisms of neuroprotection after ischemic stroke are diverse, apoptosis and autophagy can explain the destruction and regeneration of neurons relatively stable. In our study, we downregulated cleaved-caspase3 and upregulated Bcl-2 and mTOR in pMCAO through long-term stimulation of VNS, suggesting that VNS can achieve ischemic brain tissue in mice by inhibiting cell apoptosis and regulating autophagy. This has been shown to have a protective effect on the long-term neurological behavior of mice after stroke.

This study has preliminarily determined that vagal nerve stimulation therapy for stroke treatment is effective in improving neurological function, but we failed to further study its downstream signaling pathway and its key target proteins. But we will continue to further explore these in the next step. The vagus nerve stimulation method used in this study is the implantation of vagus nerve electrical stimulator. Although it is to stimulate the vagus nerve more accurately, it also causes certain trauma, which is also a limitation in this study. Yet, the research group is committed to developing noninvasive vagus nerve stimulation methods, which will further improve its clinical application.

## 5. Conclusion

The results provided in this article are the first evidence for the concept of a new strategy for using long-term VNS to achieve neuroprotection from ischemic stroke. After long-term VNS treatment on mice after cerebral ischemic stroke, we found that the neurological dysfunction of the mice was significantly improved. At the same time, histological studies found that the infarct volume of brain tissue was reduced and neuronal apoptosis was inhibited. Through changes in the expression of inflammatory proteins in brain tissue, we speculate that the protective effect of VNS on brain tissue is related to reducing cell apoptosis and regulating autophagy. Our research shows that long-term electrical stimulation of the vagus nerve can be used as a new and promising therapy for the treatment of human acute and chronic stroke. It has broad clinical application prospects and its neuroprotective mechanism is worthy of further study. Further signaling pathways and better vagus nerve stimulation methods we will continue to explore in the next study.

## Figures and Tables

**Figure 1:** Long-term VNS treatment improved neurological deficits of the mice at 7, 14, and 21 days after pMCAO. The results of quantitative analysis of mNSS (a) and adhesive removal test (b and c) were expressed as mean ± SD, *n* = 15 per group. ^∗^*P* < 0.05 vs. sham group and sham+VNS group and ^&^*P* < 0.05 vs. pMCAO+VNS group.

**Figure 2:** Long-term VNS treatment can reduce the volume of cerebral infarction in mice and increase the number of surviving neurons. (a and b) TTC-stained brain slices and quantitative analysis of the percentage of cerebral infarction volume in each group showed that compared with the pMCAO+VNI group, VNS treatment significantly reduced the infarct volume (^∗^*P* < 0.05). Data were presented as mean ± SD, *n* = 5/group.

**Figure 3:** VNS treatment decreased the apoptosis-positive cells in pMCAO. (a) FJB-positive cells in four groups of ischemic penumbra. (b) FJB-positive cell number comparison in four groups. Data were presented as mean ± SD, *n* = 5/group. ^∗^*P* < 0.05 vs. sham+VNS group and ^#^*P* < 0.05 vs. pMCAO+VNS group.

**Figure 4:** VNS treatment can reduce neuronal damage by regulating the expression of apoptosis-related proteins in the cortex around the infarct. (a) Western blots and quantitative analysis for cleaved-caspase3 and Bcl-2. (b) VNS treatment downregulated the expression of cleaved-caspase3 and upregulated the expression of Bcl-2 compared with the pMCAO+VNI group. Data were presented as mean ± SD, *n* = 5/group. ^∗^*P* < 0.05 vs. sham+VNS group and ^#^*P* < 0.05 vs. pMCAO+VNS group.

**Figure 5:** VNS treatment can reduce brain damage and protect ischemic neurons by regulating the expression of autophagy-related proteins in the peri-infarct cortex. (a–c) Western blots and quantitative analysis for mTOR, Beclin-1, and LC3-II. VNS treatment downregulated the expression of Beclin-1 and LC3II and upregulated the expression of mTOR compared with the pMCAO+VNI group. Data were presented as mean ± SD, *n* = 5/group. ^∗^*P* < 0.05 vs. sham+VNS group and ^#^*P* < 0.05 vs. pMCAO+VNS group.

## Data Availability

The underlying data supporting the results of this study are stored in the university data system and are available on request.
